# Analysis of Clinical Characteristics and Prognosis of Traumatic Brain Injury in Papua New Guinea

This article has been retracted.

**DOI:** 10.1155/2021/4948664

**Published:** 2021-12-01

**Authors:** Peng Chen, Yongbing Deng, Xing Yu, Tao Huang, Jingrui Huang

**Affiliations:** Department of Neurosurgery, Chongqing Emergency Medical Center, Chongqing University Central Hospital, Chongqing 400014, China

## Abstract

**Objective:**

To evaluate the clinical characteristics and prognosis of TBI patients from 2016 to 2019 admitted to Port Moresby General Hospital (PMGH) of Papua New Guinea (PNG) and compare the results with previous researches to analyze current clinical characteristics and prognosis.

**Methods:**

A retrospective study was performed on 389 TBI patients in Port Moresby General Hospital (PMGH) over a 48-month period (from January 2016 to December 2019). The clinical and radiographic data were collected. Patients were followed up for at least 3 months, and outcomes were assessed using the Glasgow Outcome Scale (GOS). Univariate and multivariate logistic regressions were performed to analyze the prognosis and intracranial infection of patients, as well as the effect of surgery on the prognosis of TBI patients.

**Results:**

The average age of the 389 TBI patients was 24.9 years old, and the most common age was 18-40 years old, accounting for 55.5%. The proportion of male patients was 79.4%, and the proportion of juvenile patients (≤18 years) was 30.8%. The most primary cause of injury was fighting and brawling (38.0%). At admission, patients had an average GCS score of 9.1, and patients with severe TBI accounted for 46.8%. Overall, 32.1% of the patients had a good prognosis, with a mortality rate of 13.9% (54 cases). Analyzing the relationship between surgical treatment and prognosis in 303 patients with moderate or severe TBI, there was no statistical significance. Univariate and logistic regression analyses for poor prognosis included gender, GCS, multiple injuries, Rotterdam CT scores, and intracranial infection. Univariate and logistic regression analyses for intracranial infection included GCS, open brain trauma, and postoperative drainage time.

**Conclusion:**

Despite there has been a secular trend towards reduced incidence of TBI, the prognosis of moderate or severe TBI patients who received surgery showed no significant improvement, indicating that PNG, as a backward developing country, faced a huge problem in TBI prevention and control.

## 1. Background

Traumatic brain injury (TBI) was a major public health problem worldwide and the most common inducer of death and disability in young people [1]. TBI was defined as the disruption in brain function or other evidence of brain pathology caused by an external physical force [1]. Yearly, the incidence of TBI approximately reached up to 50 million cases around the world; thus, approximately half of the global population will have an episode of TBI in their life [2].

TBI is a heterogeneous entity, reflecting several underlying macroscopic modes of injury as well as a range of mechanisms by which neuronal injury can be inflicted in differing proportions with resultant varying clinical courses [3]. Practically, the clinical severity of TBI has long been stratified according to postresuscitation Glasgow Coma Scale scores into mild (GCS 14–15), moderate (9–13), and severe (3–8) [1–3]. Severe TBI has mortality rates of 30–40% and can lead to significant physical, psychosocial, and social deficits in up to 60% of cases.

Intracranial pressure (ICP) is the most important goal-directed parameter in the clinical management of severe TBI. Raised intracranial pressure reduces cerebral perfusion risking ischemia and, when severe and sustained, brain herniation. It is of importance to maintain cerebral perfusion pressure to avoid brain ischemia because ischemia is a major contributor to unfavorable clinical outcomes following TBI.

Higher rates of morbidity and mortality are widely observed in low-income and middle-income countries, becoming a global health challenge. Previous studies have showed that the mortality rate of patients with severe TBI in low-income countries was more than twice that in high-income developed countries, and the disability rate was higher [3]. Papua New Guinea (PNG) was a low-income developing country in the South Pacific Ocean, which was short of medical resources. As early as 1996, TBI was the most common cause of traumatic death in PNG, and two-thirds of these deaths occurred before admission. TBI after admission accounted for 60% of all traumatic deaths [4]. However, in the past two decades, there are few researches on the occurrence, diagnosis, and treatment of TBI in PNG. The development of neurosurgical and talent training in PNG was not fast and satisfactory [5].

Port Moresby General Hospital (PMGH), located in the capital of PNG, was the only hospital in PNG that could provide professional neurosurgical services. Almost all patients with moderate or severe TBI were sent to PMGH. Therefore, this retrospective research collected and analyzed the data of all TBI patients treated in PMGH Neurosurgery from January 2016 to December 2019 to find out the clinical characteristics and prognosis of TBI in PNG.

## 2. Methods

### 2.1. General Information

A retrospective research on TBI patients admitted to PMGH which was located in the capital of PNG from January 2016 to December 2019 was performed. After admission, the patients were not attended by professional neurosurgeons, while brain CT examination was performed in the emergency department. Their clinical and radiographic data were collected from the hospital database.

1. Inclusion criteria: patients with TBI caused by various factors
2. Exclusion criteria: dead within 24 hours after admission; severe absence of data

### 2.2. Observation Indexes and Prognosis Assessment

#### 2.2.1. Clinical and Radiographic Variables

The clinical variables included age, gender, mechanism of TBI, Glasgow Coma Scale (GCS), multiple injuries, size of pupil, pupillary reaction, open TBI, type of brain lesion, Rotterdam CT score, surgical treatment, admission time, operation time, intracranial infection, retention of drainage tube and postoperative drainage keeping time, Glasgow Outcome Scale (GOS), etc.

Radiographic variables were collected based on brain CT at admission, including the types of TBI, Rotterdam score, and other variables.

Grades of TBI are as follows: patients with TBI were assessed with GCS on admission, 12< GCS ≤15 was defined as mild cases, 9≤ GCS ≤12 as medium cases, and 3≤ GCS <9 as severe cases.

#### 2.2.2. Prognosis Assessment

Patients were followed up by outpatient follow-up or telephone questionnaires for at least 3 months and were evaluated based on Glasgow Outcome Scale (GOS) (1 point: death; 2 points: vegetative state; 3 points: severe disability, depending upon others for daily support; 4 points: moderate disability, independent but disabled; 5 points: good recovery, resumption of normal activities, able to return to work or school). The prognosis was divided into good prognosis (GOS score 4-5) and poor prognosis (GOS score 1-3).

### 2.3. Statistical Methods

SPSS 21.0 statistical software was performed for statistical analysis. A univariate analysis for each variable was assessed using Student's *t*-test (quantitative variables) and Pearson chi-squared test or Fisher's exact test (categorical variables). A logistic regression model was developed using the univariate analysis results to identify risk factors related to poor results or intracranial infection. A *p* value less than 0.05 was considered statistically significant, and the odds ratio (OR) were calculated with 95% confidence interval (CI).

## 3. Results

### 3.1. General Patient Characteristics

According to the inclusion and exclusion criteria, 389 patients were collected with an average age of 24.9 years, the maximum age of 85 years, and the minimum age of 3 months. Seventeen cases (4.4%) were under 1 year old, 103 cases (26.4%) were between 1 and 18 years old, 216 cases (55.5%) were between 18 and 40 years old, and 3 cases (0.8%) were over 65 years old. The majority of the patients were male, accounting for 79.4% (309).

Table 1 summarizes the general clinical and radiographic data of total and young (18-40 years old) TBI patients. Fighting and brawling were the most common causes of TBI injuries in general, accounting for 38.0% with 148 cases. Among these cases, bush knife wound (92 cases) was the most common cause, followed by traffic accident injuries (34.1%). Fighting was the most common cause of injury in young patients, accounting for 62% (134 cases), which was statistically different from other TBI mechanism. There were 107 (27.5%) patients with open brain trauma and 174 (44.7%) patients with multiple injuries, while there were 70 (32.4%) young patients with open brain trauma and 86 (40%) young patients with multiple injuries. There was no significant difference between the total and young TBI patients.

The average time from injury to admission was 148.8 minutes. At admission, 212 patients (54.5%) had abnormal pupil size, 150 patients (38.6%) showed dull pupillary reaction, and 136 patients (35%) showed absent pupillary reaction. The average GCS score was 9.1, including 182 cases of severe TBI (46.8%) and 121 cases of moderate TBI (31.1%). At admission, 136 (62.5%) young patients had abnormal pupil size, 86 (39.8%) showed dull pupillary reaction, and 79 (36.6%) showed absent pupillary reaction. The average GCS score was 8.8, with 112 cases (51.9%) of severe TBI and 67 cases (31.0%) of moderate TBI. There was no statistical difference between the two groups.

The average Rotterdam score of the total patients by brain CT was 3.4, including 124 cases (31.9%) of epidural hematoma and 95 cases (24.4%) of subdural hematoma. Among the young patients, epidural hematoma was the most common, with 88 cases (40.7%). The incidence of cerebral contusion and subarachnoid hemorrhage was less (4.2%). There were statistically significant differences in types of brain lesion between the total and young patients.

Among all the patients, 225 (57.8%) patients received surgical treatment, with an average operation time of 185.6 minutes, and postoperative infection happened in 23 (10.2%) patients. Among the young patients, 136 (63.0%) patients received surgical treatment and 17 (12.5%) patients had postoperative infection.

Among all the patients, 264 patients (67.9%) had a poor prognosis after three months, while only 125 patients (32.1%) had a good prognosis. The overall mortality rate was 13.9% (54 cases), including 48 patients with severe TBI and 6 patients with moderate TBI. The mortality rate for severe TBI was 26.4% and that for moderate TBI was 5.0%. Young patients with poor prognosis accounted for 72.7% (157 cases), which was not statistically different from the total patients' data (67.9%).

### 3.2. Relationship between Surgery and Prognosis in Patients with Moderate and Severe TBI

Table 2 shows that the poor prognostic rates for moderate and severe TBI patients were 64.4% and 74.7%, respectively. We performed a prognostic analysis for moderate and severe TBI patients undergoing surgical or conservative treatment. 77 patients (63.6%) with moderate TBI received surgical treatment, while 50 patients (41.3%) had poor prognosis, showing no statistical difference from patients with conservative treatment.

118 (64.8%) severe TBI patients received surgical treatment, while 87 (47.8%) had poor prognosis after operation, which was not significantly different from that of conservative treatment.

### 3.3. Univariate Analysis of Prognosis and Intracranial Infection

Based on the good prognosis and poor prognosis, we conducted a univariate analysis of clinical and radiographic characteristics and found that gender, GCS, multiple injuries, type of brain lesion, Rotterdam CT score, and intracranial infection were statistically different between the good and poor prognosis groups. This indicated that patients with male gender, severe TBI combined with multiple injuries, subdural hemorrhage, high Rotterdam CT score, and intracranial infection were more likely to achieve poor prognosis.

For intracranial infection, we performed a univariate analysis of 225 patients undergoing surgery. We found that GCS, open brain trauma, and postoperative drainage tub keeping time after operation were statistically different between the two groups. We concluded that severe cases combined with open brain trauma and a long time (more than 36 hours) of drainage tube retention were more likely to develop intracranial infection (Table 3).

### 3.4. Logistic Multivariate Regression Analysis of Prognosis and Intracranial Infection

Logistic regression analysis revealed that factors influencing prognosis included male gender (OR: 22.2, CI: 10.5-56.6), multiple injuries (OR: 19.1, CI: 3.8-87.3), Rotterdam CT score (OR: 7.3, CI: 3.4-42.6), GCS (OR: 5.2, CI: 1.7-15.8), and intracranial infection (OR: 4.9, CI: 2.5-31.5).

Logistic regression analysis for intracranial infection revealed that factors influencing intracranial infection included open brain trauma (OR: 20.2, CI: 7.9-49.7), postoperative drainage keeping time (OR: 13.1, CI: 2.4-41.8), GCS (OR: 8.9, CI: 2.1-26.1), etc. (Table 4).

## 4. Discussion

TBI is a prominent public health and social problem in PNG. It is the primary cause of death among young people in PNG and the most common cause of death from trauma. Based on the data of PMGH, the largest general hospital in PNG, we conducted a single-center study on the clinical characteristics and prognosis of TBI in PNG, and the results were not optimistic.

When comparing this research with TBI researches of PNG in the past 30 years [4–8], we find that the following trends and features need special attention.

The first is the age composition. In the domestic research report of PNG in 2004, statistics showed that TBI patients aged 10-40 accounted for 65% [7]. In this study, TBI patients aged between 18 and 40 accounted for 55.5% of the total, with little change, indicating that TBI mainly occurred in young adults in PNG.

The second is the mechanism of TBI, mainly including violent conflicts (fighting and brawling), traffic accidents, falling accidents, and sports injuries. In the 1996 report, motor vehicle accidents (49%), assaults (32%), and falls (17%) were the most common top three mechanisms [4]. In the 2004 report, however, violent conflicts replaced traffic accidents as the main reason for TBI hospitalization, reaching 46.8%, and the proportion of traffic accidents dropped to 30.9% [7]. In this research, fighting and brawling was still the primary cause (38.0%), and analyzing young TBI patients aged 18-40 years, the proportion would increase to 62%. This showed that the problem of violence had not been effectively improved in the past decades.

We then focused on the mortality as an important prognostic indicator of moderate and severe TBI patients. In the 1996 report, the mortality rate of severe and moderate TBI patients reached 81% and 21%, respectively [4]. In the 2004 study, the mortality rate of severe and moderate TBI patients decreased to 41.2% and 8.6%, respectively [7]. In 2012, the mortality rate of severe TBI patients continued to decrease to 33.3% [5]. The results of this research on TBI patients from 2016 to 2019 showed that 32.1% of the patients had good prognosis, and the mortality was 13.9% (54 cases), with mortality of severe TBI as 26.4% and mortality of moderate TBI as 5.0%. This indicated that the overall trend of mortality of moderate and severe TBI was declining, which was inseparable from the improvement of neurosurgical treatment in PNG, especially in PMGH.

In addition to the above trends, other important features can also be analyzed from the results of this research. The mortality showed a gradually decreasing trend, but there was no significant difference compared with other low- and middle-income developing countries [9, 10]. At the same time, the poor prognostic rates of moderate and severe TBI patients were 64.4% and 74.7%, respectively. Moreover, the prognosis of moderate and severe TBI patients undergoing active operation was not significantly improved. The TBI patients with poor prognosis were very likely to suffer from severe disabilities that had great impact on life and family. We drew conclusion that in backward developing countries, moderate and severe TBIs were catastrophic events with alarming long-term consequences for individuals, families, and society as a whole.

Univariate and logistic regression analysis of poor prognosis showed that the main factors included male gender (OR: 22.2, CI: 10.5-56.6), associated multiple injuries (OR: 19.1, CI: 3.8-87.3), high Rotterdam CT score (OR: 7.3, CI: 3.4-42.6), low GCS (OR: 5.2, CI: 1.7-15.8), and intracranial infection (OR: 4.9, CI: 2.5-31.5). Univariate and logistic multivariate regression analysis of intracranial infection showed that open brain trauma (OR: 20.2, CI: 7.9-49.7), long postoperative drainage keeping time (OR: 13.1, CI: 2.4-41.8), and low GCS (OR: 8.9, CI: 2.1-26.1) were risk factors.

Consistently reported predictive factors for survival and outcome for adults with TBI include GCS, pupillary exam, imaging findings, presence of extracranial injuries, and vital signs. These variables have been incorporated into two validated models in the adult population: the Corticosteroid Randomization after Significant Head Injury (CRASH) model and the International Mission for Prognosis and Analysis of Clinical Trials in TBI (IMPACT) model. Recently, these predictive models have been shown to apply to pediatric populations with sufficient accuracy.

In our study, the average GCS score was 9.1, including 182 cases of severe TBI (46.8%) and 121 cases of moderate TBI (31.1%). At admission, 136 (62.5%) young patients had abnormal pupil size, 86 (39.8%) showed dull pupillary reaction, and 79 (36.6%) showed absent pupillary reaction. The average GCS score was 8.8, with 112 cases (51.9%) of severe TBI and 67 cases (31.0%) of moderate TBI. There was no statistical difference between the two groups. A large retrospective study that pulled pediatric patients from the National Trauma Data Bank (NTDB) showed the mortality of patients with a prehospital GCS of 3 to be 54% (*n* = 5498). This study did not remove patients with recent sedation or paralytics, which could artificially lower the mortality rate; however, patients with cardiac death on arrival were also not removed, further clouding the relevance of this mortality rate to our cohort [3, 6, 8–10]. On the whole, the results of this research showed that the treatment and prognosis of TBI patients in PNG were improved compared with ten years ago, but the data were not statistically significant. The reasons were following, first of all, poor transportation network, limited medical services in vast areas, and limited number of ambulances in rural areas in PNG; considering these factors, many urgent TBI patients were unable to be sent to PMGH in time for specialized neurosurgery treatment. The second reason was the shortage of medical facilities and resources, especially for the treatment of severe TBI patients. The whole PMGH shared 6 ICU beds and was equipped with 5 ventilators, while there were few physicians who can use ventilators skillfully. Besides, the condition of intracranial pressure (ICP) monitoring was still not available. These facts were very unfavorable for the timely treatment of patients. The final reason was the number of specialists. Currently, there were no registered neurosurgical specialists in PNG, and only two doctors could independently perform surgery for TBI, which also led to missing the best surgical time for TBI patients.

At last, we gave some suggestions on the current treatment of TBI in PNG. First of all, most of the deaths of TBI were caused by severe primary brain injury, so prevention was particularly important. The most common cause of injury in PNG in the last two decades was violent conflict (fighting and brawling), which required the joint efforts of the community, police, and government departments to maintain social order and safety, so as to effectively reduce the incidence of TBI. On the other hand, the role of the surgeon was to maximize the medical conditions and quality. From the whole process of TBI occurrence to hospitalization, the first step was to improve treatment level of prehospital and emergency department, which may further improve the prognosis of severe TBI patients. ICP monitoring in the ICU may also help prevent secondary brain injury, while postoperative intracranial infections need to be reduced by regular use of antibiotic, early and complete debridement.

PNG was also making continuous efforts to improve the treatment level and experience of neurosurgeons. Since 2005, neurosurgeons from Australia and China have been visiting PMGH regularly for guidance and teaching. Further specialist training program included regional center for short-term neurosurgery training and web-based platforms for teaching. Therefore, despite the numerous problems, it was expected that PNG can gradually improve the treatment of TBI and reduce the casualties and the burden on the family and society.

## Figures and Tables

**Table 1:** Clinical and radiological characteristics of total and young patients.

Clinical and radiological variables	Total cases (*N* = 389)	18< age ≤40 (*N* = 216)	*p* value
Age (years)	24.9 ± 7.2	—	
≤1	17 (4.4%)	—	
1< age ≤6	48 (12.3%)	—	
6< age ≤18	55 (14.1%)	—	
18 <age ≤40	216 (55.5%)	—	
40< age ≤65	50 (12.9%)	—	
65<	3 (0.8%)	—	
Male/female	309 (79.4%)/80 (3.9/1)	182 (84.3%)/34 (5.4/1)	0.15
Mechanism of TBI			
Fighting and brawling	148 (38.0%)	134 (62.0%)	<0.01
Traffic accident	121 (34.1%)	60 (27.8%)	
Fall	95 (24.4%)	12 (5.6%)	
GCS	9.1 ± 3.6	8.8 ± 3.5	
Mild	86 (22.1%)	37 (17.1%)	0.30
Moderate	121 (31.1%)	67 (31.0%)	
Severe	182 (46.8%)	112 (51.9%)	
Multiple trauma	174 (44.7%)	86 (39.8%)	0.24
Pupil size			
Normal	177 (45.5%)	81 (37.5%)	0.06
Abnormal	212 (54.5%)	135 (62.5%)	
Pupillary reactivity			
Normal	103 (26.4%)	51 (23.6%)	0.74
Dull	150 (38.6%)	86 (39.8%)	
Absent	136 (35.0%)	79 (36.6%)	
Open brain trauma	107 (27.5%)	70 (32.4%)	0.20
Type of brain lesion			
Contusion, SAH	53 (13.6%)	9 (4.2%)	<0.01
DAI	39 (10.0%)	20 (9.3%)	
EDH	124 (31.9%)	88 (40.7%)	
SDH	95 (24.4%)	47 (21.7%)	
SDH+contusion+SAH	78 (20.1%)	52 (24.1%)	
Rotterdam CT score	3.4 ± 1.5	3.1 ± 1.2	
Surgery	225 (57.8%)	136 (63.0%)	0.22
Admission time (min)	148.8 ± 23.2	—	
Operation time (min)	185.6 ± 34.6	224 ± 43.2	
Intracranial infection	23 (10.2%)	17 (12.5%)	0.35
GOS			
1, 2, 3	264 (67.9%)	157 (72.7%)	0.22
4, 5	125 (32.1%)	59 (27.3%)	

TBI: traumatic brain injury; GCS: Glasgow Coma Scale scores; DAI: diffuse axonal injury; SAH: subarachnoid hemorrhage; SDH: subdural hematoma; EDH: epidural hemorrhage; GOS: Glasgow Outcome Scale.

**Table 2:** The influence of surgery or conservative treatment on the prognosis of moderate and severe TBI.

Type of brain injury	Total patients	Treatment	Poor results	Good results	*p* value
Moderate	121	Surgical	50 (41.3%)	27 (22.3%)	0.886
		Conservative	28 (23.1%)	16 (13.3%)	
Severe	182	Surgical	87 (47.8%)	31 (17.0%)	0.674
		Conservative	49 (26.9%)	15 (8.3%)	

**Table 3:** Univariate analysis of poor prognosis and intracranial infection.

Clinical and radiological variables	Poor results (*N* = 264)	Good results (*N* = 125)	*p* value	Intracranial infection (*N* = 23)	Control (*N* = 202)	*p* value
Age (years)	25.7 ± 7.2	23.8 ± 7.6				
≤18	78 (29.5%)	42 (33.6%)	0.72	4 (17.4%)	62 (30.7%)	0.35
18< age ≤40	149 (56.5%)	67 (53.6%)		14 (60.9%)	111 (55%)	
40<	37 (14.0%)	16 (12.8%)		5 (21.7%)	29 (14.3%)	
Male/female	220/44 (5.5/1)	89/36 (2.2/1)	0.01	19/4 (4.7/1)	160/42 (3.8/1)	0.70
Mechanism of TBI						
Fighting and brawling	101 (38.3%)	37 (29.7%)	0.39	9 (39.1%)	78 (38.6%)	0.75
Traffic accident	79 (29.9%)	42 (33.6%)		9 (39.1%)	62 (30.7%)	
Fall	66 (25.0%)	29 (23.2%)		5 (21.8%)	53 (26.2%)	
GCS						
Mild	50 (19.0%)	36 (28.8%)	0.02	0	18 (8.9%)	0.02
Moderate	78 (29.5%)	43 (34.4%)		4 (17.4%)	78 (38.6%)	
Severe	136 (51.5%)	46 (36.8%)		19 (82.6%)	106 (52.5%)	
Multiple trauma	136 (51.5%)	38 (30.4%)	<0.01	15 (65.2%)	148 (73.3%)	0.41
Pupil size						
Normal	112 (42.4%)	65 (52%)	0.08	10 (43.5%)	90 (44.6%)	0.922
Abnormal	152 (57.6%)	60 (48%)		13 (56.5%)	112 (55.4%)	
Pupillary reactivity						
Normal	62 (23.5%)	41 (32.8%)	0.09	5 (21.7%)	54 (26.7%)	0.85
Dull	102 (38.6%)	48 (38.4%)		10 (43.5%)	78 (38.6%)	
Absent	100 (37.9%)	36 (28.8%)		8 (34.8%)	70 (34.7%)	
Open brain trauma	78 (29.5%)	29 (23.2%)	0.19	19 (82.6%)	88 (43.6%)	<0.01
Type of brain lesion						
Contusion, SAH	27 (10.2%)	26 (20.8%)	0.04	0	0	0.90
DAI	24 (9.1%)	15 (12%)		0	0	
EDH	88 (33.3%)	36 (28.8%)		5 (21.7%)	48 (23.8%)	
SDH	67 (25.4%)	28 (22.4%)		8 (34.8%)	61 (30.2%)	
SDH+contusion+SAH	58 (22.0%)	20 (16.0%)		10 (43.5%)	93 (46.0%)	
Rotterdam CT score	3.8 ± 1.5	3.1 ± 1.7	0.01	3.3 ± 1.3	3.5 ± 1.5	0.93
Surgery	148 (56.1%)	77 (61.6%)	0.30	—	—	
Admission time (min)	162 ± 27.2	129 ± 21.7		—	—	
Operation time (min)	180.6 ± 30.1	192.6 ± 37.6		196.8 ± 34.6	183.6 ± 36.4	
Intracranial infection	18	5	0.04	—	—	
Drainage tub	—	—		20 (87.0%)	166 (82.2%)	0.57
Drainage tub keeping time (h)	—	—		37.2 ± 17.6	30.4 ± 16.3	0.01

GCS: Glasgow Coma Scale scores; DAI: diffuse axonal injury; SAH: subarachnoid hemorrhage; SDH: subdural hematoma; EDH: epidural hemorrhage.

**Table 4:** Logistic multivariate analysis of poor prognosis and intracranial infection.

Variables	SE	Wals	*p* value	OR	95% CI
Poor results					
Male	0.4	56.7	<0.01	22.2	10.5-56.6
GCS	0.6	8.2	0.03	5.2	1.7-15.8
Multiple trauma	0.8	12.7	<0.01	19.1	3.8-87.3
Rotterdam CT score	0.7	4.8	0.03	7.3	3.4-42.6
Intracranial infection	0.6	8.3	0.03	4.9	2.5-31.5
Intracranial infection					
GCS	0.5	9.3	0.03	8.9	2.1-26.1
Open brain trauma	1.1	6.4	<0.01	20.2	7.9-49.7
Drainage tub keeping time (h)	0.8	5.3	0.01	13.1	2.4-41.8

GCS: Glasgow Coma Scale scores.

## Data Availability

The data used during the present study are available from the corresponding author upon reasonable request.
